This article has been retracted.

# Deep Intelligence-Driven Efficient Forecasting for the Agriculture Economy of Computational Social Systems

**DOI:** 10.1155/2022/2854675

**Published:** 2022-09-27

**Authors:** Xuelan Li, Xiao Li, Jiyu Jiang

**Affiliations:** ^1^School of Management, Anhui Science and Technology University, Bengbu, Anhui 233030, China; ^2^Faculty of Metallurgical and Energy Engineering, Kunming University of Science and Technology, Kunming 650093, China; ^3^School of Economics and Management, Anhui Agricultural University, Hefei, Anhui 230036, China

## Abstract

In the vision of smart cities, everything is highly connected with the aid of computational intelligence. Therefore, the cyber-physical society has been named a computational social system for a long time. Due to the high relation with vast populations' national livelihood, agriculture will still serve as a core industry in the national economy. As a result, this study focused on an efficient forecasting method for the agriculture economy. In recent years, the conception of deep intelligence has received overall prevalence in academia because of its excellent performance in implementing intelligent information processing tasks. Hence, this paper utilized deep intelligence driven by neural networks and managed to investigate an efficient prediction method for the agriculture economy of computational social systems. To fit the time-series forecasting scene of the long-term development of the agriculture economy, the convolutional neural network model is slightly improved by revising its parallel structure into the recurrent format. Finally, simulations on realistic datasets are carried out to evaluate the proposed forecasting method.

## 1. Introduction

Agricultural economic development is related to people's livelihood issues and has an essential impact on the economic development status of industries related to the farm economy. Therefore, a good development trend in the agricultural economy is vital for promoting stable economic growth. The output of agricultural products is an important indicator to reflect the farm economy [1]. The information about the supply and demand of agricultural products has become more complicated. Effective forecasting of agricultural production can better enable agrarian producers to understand information about agricultural production, take appropriate measures promptly for possible problems in the process of the farm output and provide solutions suitable for the development of the farm economy regarding agricultural production inputs, thus promoting the smooth operation of the farm market [2]. In rational planning of agricultural production, it is necessary to quantitatively analyze the main factors affecting agricultural production and predict the trend of the farm output. As a direct time series forecasting method, the ARIMA model is widely used in forecasting agricultural production [3]. Gray forecasting is also a standard method for agricultural yield forecasting due to the characteristics of the gray forecasting model with low data requirements. Model averaging is a more popular method to solve the model selection uncertainty problem and is one of the critical ways to improve the forecasting level [4]. Therefore, applying the model averaging process to forecasting agricultural yield can effectively reduce the forecasting error of agricultural work [5]. Based on the ARIMA model, gray prediction model, and model averaging method, three different ways to predict agricultural yield get different results; comparing and analyzing the prediction level of pastoral work under other prediction models provides an effective prediction method for more accurate prediction of agricultural output, which will give solid suggestions for the farm development plan [6].

Deep learning techniques have made impressive achievements. Technology development has become more mature, with extensive applications in various fields, such as data mining, machine translation, natural language processing, facial recognition, target recognition, etc. [7]. With the development of the Internet, computer vision used in deep learning provides the possibility to solve problems such as crop diseases and is widely used in agriculture [8]. Advanced computing techniques such as artificial neural networks, recurrent neural networks, and convolutional neural networks have led to various nondestructive algorithms and methods [9]. The accuracy of classification using such models has surpassed that of humans. Le Net was the first convolutional neural network in the traditional sense [10]. Alex Ne emerged in the Image Net visual recognition challenge in recent years. After Alex Net, convolutional neural networks developed rapidly, and neural networks such as VGGNet, Google Net, and Res Net emerged [11]. With the deepening of the network model structure, the accuracy of wide image recognition is getting higher and higher, so the application in disease recognition of crops is becoming more widespread. There are numerous methods of deep learning for disease recognition of crops [12].

Traditional economic forecasting models mainly include time series analysis, correlation analysis, gray forecasting, and some combination forecasting methods. Most use linear models, all of which have specific forecasting abilities and shortcomings [13]. Because the economic system is a complex giant with many internal influencing factors and strong time-varying, coupling, and nonlinear characteristics, it is challenging to model and predict the financial system with many factors [14]. Artificial neural networks have received increasing attention from researchers since the rise of artificial intelligence in the 1980s and have become a current research hotspot. It is a mathematical model that simulates the human brain by an engineering based on biology, with good nonlinearity, self-organization, fault tolerance, and parallel processing ability [15]. In the past decade, researchers have been studying artificial neural networks. Many improvements have been made, and the performance of artificial neural networks has been optimized and used in many fields. The error backpropagation (BP) neural network algorithm is a neural network model currently used more often. Still, it has the defects of slow training speed, easy falling into local extremes, and easy overfitting, improving the convergence speed and having better nonlinear mapping ability than the CNN neural network model [16]. In this paper, we start from two key aspects of agricultural economic time series forecasting by the convolutional neural network: time series analysis technique and forecasting tool selection. By improving the critical elements of time series analysis, such as model order fixing, variable hoof selection, and training sample selection, and selecting suitable forecasting tools by combining the characteristics of agricultural economic time series data, we aim to improve the prediction accuracy of agricultural economic phenomena such as grain yield and gross agricultural output index by a large margin. The aim is to improve the prediction accuracy of agricultural economic phenomena such as grain yield and gross agricultural output index and provide valuable references for prediction in other fields of agricultural science.

## 2. Related Works

Information technology is one of the main channels to promote rapid economic development. The degree of information technology development is also an indicator of total national power; information technology is widely used in various industries [17]. Another representative macro-level measurement method is the Borat method, which classifies the information industry to get the information sector and uses the information sector gross product to measure the development level of the information economy. The second level is the information index algorithm, proposed by economist Rambaccussing and Kwiatkowski, which selects a benchmark indicator and weights the constructed indicator with the benchmark indicator to obtain information development [18]. Nowadays, most of the literature and the actual measurement of agricultural informatization are based on the information industry GNP algorithm, the information index algorithm, and the Borat measurement method, and variants are made [19]. The methods commonly used by scholars at this stage are the index evaluation method and the Borat method. The relevant literature studies, and on this basis, he concluded that the standard, comprehensive evaluation methods for agricultural informatization are mainly principal component analysis and DEA. Sava et al. constructed a BBC model for analysis by quantitative analysis of rural informatization using the DEA method [20]. The research used a self-selected evaluation system of agricultural informatization investment and output efficiency indicators for the empirical study. Malik et al. also chose the same DEA method, but the model selection differed [21]. Aparicio et al. chose the hierarchical analysis method to construct an evaluation system of the agricultural informatization level indicators and used the coupling degree to analyze the relationship between farm informatization and the farm economy [22].

The development of agriculture has a history of several thousand years, and agriculture is an essential support for the governance of the country and the harmonious and stable life of the people and is the foundation and guarantee for the steady operation of the whole economic and social system [23]. In a study related to measuring the high-quality development of the agricultural economy, Medeiros et al. measured the effect of rural modernization in each country in terms of the level of agricultural development, the group of rural infrastructure construction, the level of pastoral development support, and the level of sustainable agricultural development, and quantitatively analyzed the status of rural modernization development of the observed sample [24]. The study found that most countries had uneven and unbalanced development levels, except for individual countries. In terms of the strength of the level of agricultural support and protection, the countries with more backward economies are more significant than those with more leading economies, and the resource and environmental conditions are relatively better in economically backward areas.

All countries are classified through the comprehensive index situation, and related policies and suggestions are put forward. At the same time, Colombo and Pelagatti constructed a complete evaluation system from the main characteristics of the high-quality development of the agricultural economy, and through the analysis of the data model, it is concluded that the critical factors affecting the high-quality development of the farm economy are agricultural, natural resource elements, and regional economic development level, and the level of high-quality development of the rural economy in the eastern region is higher and ahead of other areas; the development of each region has different advantages and disadvantages; the grain-producing central areas have a lower level of agriculture; the level of high-quality economic development was quiet and still needs to be improved [25]. We should choose the direction of high-quality development of the rural economy according to local conditions, the disadvantage factors of high-quality development of the agricultural economy in each region and the advantage oriented planning of each area, lead the high-quality development of the rural economy in the eastern part with green development and innovation development; enhance the development of unique agricultural products in the western region and increase the infrastructure construction to promote high-quality development; focus on the security and safety of food crops in the prominent grain-producing areas and promote the coordinated, high-quality development. Wang focuses on the concept of sustainable development and takes the sustainable development of the whole system as the direction of choice, establishes the five indicators of population, society, economy, resources, and environment, and builds the evaluation system of sustainable agricultural development with the framework of these indicators [26]. The observation sample is selected from the prominent grain-producing areas. Scholars have also conducted much research work using artificial neural networks in economic system forecasting. They were among the first scholars to apply neural network methods to financial forecasting and analyzed neural network methods compared to traditional methods.

## 3. A Deep Intelligence-Driven Approach to Agricultural Economy Forecasting for Computational Social Systems

### 3.1. Deep Intelligence-Driven Modeling of Computational Social Systems

Social computing has made a significant contribution to the era of notification. Only professionals with a certain level of computer knowledge could use computers in the past. Still, since the emergence of social computing, some users with only rudimentary network experience can use the Internet at will because social computing has lowered the requirements for using computers. This allows the average user to use the Internet freely without the limitations of technology, fully express their talents, and share resources online. This feature is already relatively evident in the business world, such as the decision by some companies and organizations to shift market dominance to consumer networks. Numerous lightweight and useful open-source software also provide a platform for grassroots innovation, which will not only pose a threat to traditional software developers but may even establish new business models. Drawing on these experiences, recognizing and adapting to these changes in the archival digitization process can enable archivists to address better the challenges facing by the existing archival digitization model, seize all possibilities for developing archival digitization and be well prepared for achieving a higher level of digital archival management.

Along with in-depth research on technologies such as knowledge management and intelligent deep analysis, deep intelligent systems based on the knowledge level have become an indispensable part of the development of artificial intelligence. Deep intelligence systems mainly use a combination of the deep QA framework structure and the knowledge graph inference to process problems through cascading collaborative processes, significantly improving system framework extension and intelligent inference analysis. An important application of deep learning, also known as deep neural network (DNN) in NLP, besides word embedding to characterize the semantics of words, which is another vital advancement is the use of CNN to calculate the similarity between sentences and the use of RNN or LSTM to do the encoding and decoding of sentences. Classified according to the neural network propagation method, CNN is a non-fully connected feedforward neural network that connects with the next layer through a weight-sharing strategy, which can effectively save the training overhead of model parameters and is a core technology for computer vision systems. Because of its powerful ability to capture local features, CNN performs well in image recognition tasks and many tasks in NLP. Convolutional neural networks can usually be divided into input, convolutional, sampling, connection, and output layers. A convolutional neural network is a variation of the development branch of neural networks.

The weight parameter assignment structure, which simplifies the complexity of the network, allows image data to be used directly as layer inputs, avoiding the process of complex image data preprocessing. The convolutional neural network processing of 2D image data is equivalent to a special multilayer perceptron. In the quantification process, the contours are drawn first and then divided into different levels for the indicators that can be directly quantified, such as ground stress value, vertical strain gradient, and ground temperature gradient. The rating comparison method divides the levels according to the index's planar distribution characteristics that cannot be quantified directly. This perceptron model has a high linear invariance, which ensures that the information does not change during translation, scaling, tilting, or other forms of deformation of the expressive feature information dimension data. The discussion of convolutional neural networks focuses on implementing convolutional operations to train multilayer network structures using accurate input image data [27]. It can combine spatial information of image data to learn and extract image features adaptively. The root of deep learning is the iterative update type convolutional neural network, which extracts and integrates data feature information through the lowest level of input image data and iterates into different levels of operations sequentially; each iteration has corresponding digital filters to realize the training data reading function and finally obtains the predicted result output. From the surface of the hierarchy, the convolutional neural network is a planar linear structure, each layer consists of two-dimensional image information operations built up, and the functional unit layers act independently of each other at each step stage, without the influence of cross-information between each other, as shown in Figure 1.

CNN is like a standard fully connected neural network. Still, the main difference is the network components, consisting of a convolutional layer, a pooling layer, and a fully connected layer. The convolutional layer contains the convolutional operations and the RELU activation function. CNN takes the original image data through processes such as convolution and pooling. It then uses a backpropagation algorithm to train the model and converts it into a feature vector with semantic similarity to the original image.

(1) Convolutional layer: The convolutional layer is generally located behind the network's input layer and is one of the essential parts of CNN. Convolutional computation is to scan the input data using convolutional kernels and then combine the data with local weights to obtain the corresponding feature maps. Convolution kernels of different sizes are different feature extractors that extract local features in multiple directions of the input image. Suppose the *i* input feature map of the convolutional layer is *n*_(*i*)_, and its corresponding *j* feature map output is *fout*_(*j*)_, whose expression is
  (1) $$\begin{array}{c} \left.{f\text{ou}}_{\left(j\right)}=\underset{i=1}{\sum }\left(\frac{fin\left(i-1\right)}{w_{ij-1}}\right.+b_{j}\right)\text{.} \end{array}$$
(2) Pooling layer: Generally, a pooling layer is designed between multiple convolutional layers to further process the feature map from the convolutional layer, effectively reducing the feature map's size and filtering out the critical feature information. Suppose the size of the feature map does not change during the training process of the convolutional neural network. The number of operations in the convolutional and fully connected layers will be much more aggravated, resulting in slow training and even complex network convergence. Using a pooling layer vastly reduces filters of some useless or less useful features, significantly reducing the redundancy of elements in the network. Maximum pooling means that the pooling kernel takes the maximum of its feature points in a neighborhood selected by the sliding window operation.
(3) Fully connected layer: The fully connected layer is an ordinary neural network layer, unlike the local perception of the convolutional layer, where each neuron is fully connected to each neuron in the next layer. The number of operations is more significant, which can significantly improve the fitting ability of the network. Generally, after several convolutional layers, pooling layers, and activation functions, a fully connected layer is added at the end of the convolutional neural network to enhance the fitting ability of the whole network as well as to get the output of specified length, i.e., after the fully connected layer, the fully connected production of the last layer is set to the size of the final output. The equation for the fully connected layer is as follows:
  (2) $$\begin{array}{c} R_{f}=\sum \frac{\sqrt{w-1}}{\sqrt{x+b}}\text{.} \end{array}$$
(4) Loss function: The loss function is an essential function in deep learning neural networks, which refers to the goal of the training network, that is, the purpose of training. Different loss functions are chosen for other problems. For the regression problem, Euclidean loss can be selected as the loss function of BP, i.e., CNN is to reduce the number of parameters needed to train the neural network by the perceptual field and weight sharing.
Too many BP weights means too much computation.
  (3) $$\begin{array}{c} \left.\text{Euclideanloss}=\underset{i=1}{\sum }\left(\frac{y_{i}^{n}}{\sqrt{y_{i}+2}}\right.\right)\text{.} \end{array}$$
The meaning of Euclidean loss is the mean square error between the actual output and the network output, which is the most common loss function when doing regression training. The absolute error function of the loss function for regression problems, such as:
  (4) $$\begin{array}{c} Absoluteloss=\underset{i=1}{\sum }\frac{\sqrt{y_{i}^{n}+y_{i}}}{n-1}\text{.} \end{array}$$
(5) Whether it is a convolutional or fully connected layer, the network is computed by multiplying the weights plus the bias, and the whole process is linear. Suppose a nonlinear activation function is not added. In that case, the network will not be able to handle nonlinear problems, even simple heterogeneous issues cannot be solved, and the deep network structure will be meaningless. Neural networks use the activation function to improve the nonlinear fitting ability. The activation function is usually added after the pooling and fully connected layers in convolutional neural networks. There are several standard activation functions: the classical sigmoid activation function and its variant tan*h* activation function, the newer RELU (Rectified Linear Units) activation function, and its variants p-RELU, and LEAKY-RELU. Prone to gradient disappearance or gradient explosion, RELU improves this problem by its sparsity, i.e.,
  (5) $$\begin{array}{c} FRelu\left(x\right)=\sum \max\left(\sqrt{x-1}\right)\text{,} \end{array}$$
  (6) $$\begin{array}{c} Fsigmoi\;d\left(x\right)=\int \frac{x-1}{\sqrt{e^{x}-1}}\text{.} \end{array}$$

### 3.2. Model Design of the Agricultural Economy Forecasting Method Based on the Convolutional Neural Network

Financial forecasting is the application of forecasting theory and forecasting methods to economic systems. The development of the economy is generally nonlinear, dynamic, and uncertain. Economic growth factors are complex: resource structure, industrial action, transportation and logistics, capital introduction, talent introduction, policy, etc. They are closely related, making the economic system a complex giant system. In addition to the completeness of data, the chosen forecasting method's scientific and rationality also affect the forecasting results to a large extent [28]. The flow chart of financial forecasting methods is shown in Figure 2. By the nature of forecasting, there are qualitative and quantitative forecasts. Qualitative forecasting is used when it requires only a general understanding of the forecasted object, a description of its tendency to change, and a judgment of its probability or improbability of occurrence. Quantitative forecasts are used when the future values of some economic indicators are projected from the known values of others, and the likelihood of reaching these values is stated. In this case, the importance of the forecasted variables is expressed as a single value and is called point-value forecasts; the values of the forecasted variables have a range within the interval between the upper and lower limits and are called interval forecasts.

The network's input must be determined first when using CNN for agricultural economic forecasting. For the *y*-*y* model, the time window is generally selected using trial-and-error to determine the information of the network; for the *u* − *y* model, the variables with a mutual relationship number more significant than a threshold with the output are first selected as the variables of interest using the CCA algorithm, and then the time window is determined using the time lag information derived from the CCA algorithm; similarly, the inputs of the *u* − *e* and *uy* − *y* models can be determined. For the network structure of the CNN prediction model of the *y*-*y* model, considering the characteristics of the input dimension, unlike the traditional image processing methods that use a square convolutional kernel size, a long strip-shaped convolutional kernel, and a pooling kernel size can be selected, and the specific steps are as follows:

  STEP 1: Analyze the data and select the appropriate time window using the trial-and-error method.
  STEP 2: Using several convolutional and pooling layers with long strip size convolutional kernels and pooling kernels, the input width is reduced to a smaller value, *W* − 1.
  STEP 3: Add a fully connected layer to get the network output.
  STEP 4: Train the model and adjust the network structure according to the effect.

For the *u* − *y* and *u* − *e* models, the CNN structure is designed similarly.

When there is only one correlated variable, the network is designed similarly to the *y*-*y* model, except that the CCA algorithm is selected for determining the time window. Considering the case of multiple correlated variables, the variables with the number of interrelationships greater than a threshold are first chosen as the correlated variables using the CCA algorithm [29]. Then the maximum time lag *T* of these correlated variables is selected and multiplied by the correction factor *k* as the value of the time window length *s*. For the network structure, this paper proposes to change the input width to 1 by selecting a rectangular convolutional kernel with a width equal to the input dimension in the first convolutional layer. For the case of *n* correlated variables with a time window length of *s*, the size of the convolutional kernel utilized firstly changes the input width to 1. It then uses the CNN design steps of the *y*-*y* model to design. For this purpose, the steps to create *u* − *y* and *u* − *e* type network structures are as follows:

  STEP 1: Analyze the data and using the CCA algorithm, select the most significant time lag *t* of these correlated variables and multiply the correction factor *k* as the value of the time window length *s*.
  STEP 2: The input width is changed to *i* in the first convolutional layer using a convolutional size kernel.
  STEP 3: The subsequent network structure design is carried out using the CNN design steps of the *y*-*y* model. *u* − *y* and *u* − *e* method structure diagrams are shown in Figure 3.

For the *guy* − *y* method, the feasible idea is to use *y* and you equally as input and adopt the network structure design of *u* − *y* and *u* − *e*. The steps of CNN offline training are to first obtain historical data from the production process and analyze and preprocess the data. The preprocessing includes outlier rejection, data normalization, and CCA to get correlation and time-lag variables. Then, the CNN network structure is designed according to the characteristics of the data, and the processed data are fed into the network for training. After reaching the number of training iterations, the results are checked to see if they meet the requirements. If not, the network structure is adjusted and retrained until satisfactory results are achieved. Because of the dynamic nature of economic phenomena, their development is influenced by many uncertainties, so errors are inevitable. However, we can control the error within a reliable range using model parameter adjustment and other means to ensure the validity of the results. Performing time prediction online is the process of CNN forwarding. First, the production process of getting real-time data from DCS and normalizing the data in the same way as in training preprocessing, then the normalized data is sent to the convolutional neural network for prediction to get the output. Then the result is back-normalized and cycled to wait for the next moment of incoming data.

The performance of convolutional neural networks in time series prediction and causality prediction in two cases: sudden changes in the original data and drastic changes in the original data. One unit-year is taken in the input layer, one unit of total production is taken in the output layer, three teams are taken in the implicit layer, and the original data set is prepared in any order. All the original data are learned, and a CNN network model is built. At the same time, a gray series prediction model GM (1, 1) is made for the total yield series of food crops. Regarding fitting accuracy, the maximum relative error of GM (1, 1) is 23.3%, while the maximum relative error of the CNN network is only 4.5%. In terms of fitting accuracy, the calculation result of the GM (1, 1) model is exponentially decreasing, which is unsatisfactory for future forecasting. There are sudden changes in the past. It cannot be said that there will be sudden changes in the future, so let's look at the causality prediction again. Applying the convolutional neural network model, the input layer takes one unit-the sown area, the implicit layer takes one layer of three teams, and the output layer takes one unit-the yield. All the historical data are learned, or several sets of data are arbitrarily divided from the original data as “test data,” while other data sets are used as “training data.” At the same time, the GM (1, 2) model is applied to establish the response equation between total grain crop yield and sown area, which could be used for prediction. Given the same inputs, the resulting prediction results are shown in Figure 4.

## 4. Analysis of Results

### 4.1. Model Analysis of Agricultural Economic Forecasting Methods

The agricultural economy is a general term for economic relations and economic activities in agriculture: financial activities, production, exchange, distribution, and consumption links. Due to the limitation of science and technology, the ancient agricultural economy was kept in the state of slash-and-burn farming, which lasted for thousands of years before the industrial revolution. The rapid development and breakthroughs in science and technology subsequently led to the application of more advanced scientific and technological achievements and management methods to the development of agriculture, facilitating the transformation of traditional agriculture into agricultural modernization [30]. Countries are paying more and more attention to the development of the farm economy through its macro-control and policy guidance to promote further the steady and sustainable development of the agricultural economy. This paper constructs an agricultural economic forecasting model based on the convolutional neural network model. Estimating in advance may produce errors, and the forecasting method should be tested before use. This paper constructs several standard regression models using the sclera library for performance comparison based on agricultural economic forecasting data. And the prediction results are plotted against the actual values as line graphs. The comparison graph of the prediction effect of multiple regression models for the dataset is shown in Figure 5.

SVR, SVR-CAR, and GS-RSR-SVR were implemented and validated with the self-programmed MATLAB program call toolbox LIBSVM2.9 [7], all of which selected the radial basis kernel as the kernel function (the radial basis kernel exhibits a better generalization promotion performance than other kernel functions on most data sets, while it is a typical local kernel function that meets this paper's GS regionalization variable analysis requirements). Based on the one-step prediction method, the other reference models MLR, CAR, ARIMA (for data *A* and data *B*: *p* = *d* = *q* = 2; for data *C*: *p* = *d* = *q* = 4), and BPNN (the number of implied layers is 1, the number of nodes in the indicated layer is 2*∗n*+1 (*n* is the number of independent variables) the number of input nodes is the number of independent variables, the training rate is 0.1, the allowable error is 0.0001, the maximum number of iterations is 1000) are given by DPS6.55.

Agricultural economic forecasting using a convolutional neural network model derives the requested forecast values from a nonlinear function trained on sample data. However, since different economic indicators vary widely with strong and weak correlations, selecting appropriate influencing indicators as inputs to the neural network is particularly important in model prediction. In this paper, the 39 collected indicators are analyzed for their characteristic importance, and the indicators are selected scientifically and objectively using a scientific method for the reasonableness of the predictors. The Pearson correlation coefficient heat map can show the correlation between two features. The correlation analysis of agricultural economic data features is shown in Figure 6.

As a critical part of the model prediction, the prediction model directly affects the accuracy of the subsequent steps. A CNN-based prediction model for time lag analysis of correlated variables is used. The prediction model begins by determining the input range. The model prediction control incorporates the past inputs of the variables and the future values within the control step as part of the inputs to the prediction model. Based on the information and outputs and their time windows, the CNN prediction structure for this system is built using the *uy* − *y* model. Using the MPC algorithm, subsequent multi-step predictions now *P* are required. At *P* = 5, five CNN prediction models need to be trained. In rolling optimization, each iteration must be computed separately for each model. The computational effort grows proportionally with the prediction step *P*. Therefore, 5 prediction steps are simultaneously considered in one CNN model. The number of outputs of the last CNN fully-connected layer is set to 5, and the Euclidean loss is used to compute the training so that the sum of squared errors of the 5 predictions is minimized. The prediction profiles in the test set are shown in Figure 7.

To achieve the relative optimum of optimization performance and control performance under a long cycle, based on the OEST-EMPC control strategy, a cyclic economic model predictive control strategy applicable to the optimization control process of the long cycle is proposed. The finite-time OEST-EMPC is designed to estimate the switching time online within the finite-time 6 so that the system's overall performance is optimal to ensure both the economic performance improvement and the control target. After the system reaches the control target, it remains in the control mode until the state is “perturbed.” The above process is a single cycle, cyclic in the long-period control process. The system is controlled periodically and optimally. Whenever the system is “perturbed,” the time is reset to zero, and a new cycle is started. This not only balances the economic and control performance but also solves the problem of free switching between optimization and control modes and extends the limited terminal time to infinite time, which is more in line with the actual production requirements.

### 4.2. Implementation of Agricultural Economic Forecasting Method Based on the Convolutional Neural Network

The classification performance of the algorithmic model, as demonstrated on the experimental dataset, is analyzed. Different hyperparameters are fine-tuned for other methods, and many experimental parameters are tested to find the most suitable algorithmic model. For the agricultural economic forecasting task, we constructed a Conv GRU convolutional time series neural network model capable of learning temporal and spatial features to explore the feasibility of using long-term historical agricultural economic information and data for yield forecasting based on deep learning methods [31]. The network uses extensive data from remote sensing of crops over many years as input, takes complete account of the temporal variation characteristics of variables, and achieves agro-economic forecasting by capturing abnormal changes in variables during the growth period. We also highlight the superiority of the proposed algorithm by comparing it with a multiple linear regression model using a small amount of data with other multiple neural network fitting models based on the CNN neural network algorithm. In addition, the actual data are estimated from the area statistics combined with the predicted values. The expected results with the agricultural economic values are shown in Figure 8.

After analyzing the mechanism of action of agricultural economic forecasting, we next scrutinize and further measure the interaction between the two from the perspective of nonlinear transfer, using the CNN model constructed above, the growth rate of gross agricultural output (TAGR) and the time series of the fluctuating component of GDP growth rate (TCYCGDP) data. Before starting the econometric analysis, based on various methods such as ADF test, PP test, and KPSS test, we specifically investigate the smoothness of the fluctuating components of the growth rates of gross agricultural value and GDP, which can verify the hypothesis we put forward in the previous section when constructing the nonlinear CNN model, that the analysis of the time series should satisfy the requirement of smoothness. The test results show that both series are smooth at the 5% significance level, and both are first-order single integers at the 1% significance level. Based on the above tests, we use AIC, HQ, SC, and other information criteria, as shown in Figure 9, to calculate AIC, HQ, and SC values for each model-specific setting form. In this process, we consider various cases, i.e., nonlinear CNN models with the number of zones of 2 (*M* = 2) and 3 (*M* = 3) and lag orders from −1 to 1 in that order. After comparison, we can see that we obtain the smallest of the three values using the CNN model, which means that using the CNN model can play a reliable role in drawing valid conclusions.

According to the comparison, for data 1, the AIC value is much lower than that of the comparison model; similarly, for data 2, the AIC value is also the lowest, and the minimum average error of the prediction results indicates that the model has the highest prediction accuracy and can well describe the changing pattern of agricultural economic time series data. It can be seen that the prediction errors of the linear models MLR, CAR, and AMRA are greater than those of the nonlinear models and the prediction models proposed in this paper, indicating that the agricultural economic time series are with nonlinear change patterns and the use of linear models to model and predict them, which is fundamentally unfeasible and has the defect of acceptable prediction accuracy; In contrast, the prediction accuracy of the BPNN1 model without chaos analysis is lower than that of CNN, the prediction model of the neural network indicates that without chaos analysis of agricultural economic time series and phase space reconstruction, it cannot accurately and comprehensively describe the nonlinearity, chaos, and time lag of agricultural economic time series.

## 5. Conclusion

The development process of modern agriculture has entered the level of scientific management, and scientific and technological innovation is an important driving force for the conversion of old and new dynamics of agricultural development and supply-side structural reform; the application of agricultural economic forecasting models and methods has laid the foundation for the realization of scientific and technological agrarian development. Compared with CNN neural networks and vector autoregressive VAR models, DBN deep learning methods have a better forecasting performance, and the mean relative error of their forecasting results has comparative advantages; due to the introduction of pretraining, the deep learning method has faster convergence speed and higher convergence accuracy in the training phase; in the case of limited labeled training samples, the convolutional neural network method can improve the prediction performance of the system by pretraining with unlabeled samples. Still, with many unlabeled samples, the prediction performance of the convolutional neural network method has limited degradation. The convolutional neural network method has better generalization ability than the supervised learning method of the BP neural network, which requires many labeled samples. The results show that the convolutional neural network-based agricultural economic forecasting method improves the accuracy of agricultural financial forecasting and reduces the forecasting error.

## Figures and Tables

**Figure 1:** Layer diagram of the convolutional neural network.

**Figure 2:** Flow chart of the economic forecasting method.

**Figure 3:** Structure of *u* − *y* and *u* − *e* methods.

**Figure 4:** Total production forecast for future years.

**Figure 5:** Comparison of prediction effects of multiple regression models for the data set.

**Figure 6:** Correlation analysis of agricultural economic data characteristics.

**Figure 7:** Prediction graphs in the test set.

**Figure 8:** Predicted results and agricultural economic values.

**Figure 9:** Comparison of AIC values, HQ values, and SC values for the specific setting form of the model.

## Data Availability

The data supporting the conclusion of the article are shown in the relevant figures and tables in the article.
